RETRACTED

# Ultrasonic Elastography Combined with Human Papilloma Virus Detection Based on Intelligent Denoising Algorithm in Diagnosis of Cervical Intraepithelial Neoplasia

**DOI:** 10.1155/2021/8066133

**Published:** 2021-12-26

**Authors:** Lu Sun, Xiuling Shan, Qihu Dong, Chong Wu, Mei Shan, Hongxia Guo, Rui Lu

**Affiliations:** Department of Obstetrics and Gynecology, Shuyang Hospital of Traditional Chinese Medicine, Shuyang, 223600 Jiangsu, China

## Abstract

The aim of this research was to study the application of ultrasonic elastography combined with human papilloma virus (HPV) detection based on bilateral filter intelligent denoising algorithm in the diagnosis of cervical intraepithelial neoplasia (CIN) and provide a theoretical basis for clinical diagnosis and treatment of CIN. In this study, 100 patients with cervical lesions were selected as research objects and randomly divided into control group and experimental group, with 50 cases in each group. Patients in control group and experimental group were diagnosed by ultrasonic elastography combined with HPV detection. The experimental group used the optimized image map of bilateral filter intelligent denoising algorithm for denoising and optimization, while the control group did not use optimization, and the differences between them were analyzed and compared. The diagnostic effects of the two groups were compared. As a result, the three accuracy rates of the experimental group were 95%, 95%, and 98%, respectively; the three sensitivity rates were 96%, 92%, and 94%, respectively; and the three specificity rates were 99%, 97%, and 98%, respectively. In the control group, the three accuracy rates were 84%, 86%, and 84%, respectively; the three sensitivity rates were 88%, 84%, and 86%, respectively; and the three specificity rates were 81%, 83%, and 88%, respectively. The accuracy, sensitivity, and specificity of experiment group were significantly higher than those of control group, and the difference was statistically significant (*P* < 0.05). In summary, the bilateral filter intelligent denoising algorithm has a good denoising effect on the ultrasonic elastography. The ultrasonic image processed by the algorithm combined with HPV detection has a better diagnosis of CIN.

## 1. Introduction

Cervical intraepithelial neoplasia (CIN) refers to the general name of precancerous lesions related to cervical invasive cancer. There are cervical atypical hyperplasia and cervical carcinoma in situ. In recent years, there are a large number of relevant reports at home and abroad, which have a preliminary understanding of the continuous development process of cervical cancer [1]. The cause of cervical intraepithelial lesions is the persistent infection of high-risk human papilloma virus (HPV), of which HPV16 is still the most common HPV type. About one million women in the United States suffer from cervical epithelioma like lesions. Women of any age may suffer from the disease, but it is the highest among women aged 25~35 [2]. At present, although it was confirmed that persistent HPV infection is the clear cause of cervical intraepithelial lesions and cervical cancer, HPV infection does not necessarily lead to cervical intraepithelial lesions or cervical cancer [3, 4]. Most young women, especially those under the age of 21, can have the HPV infection cleared within 8 months or have the viral load reduced to negative level. In this kind of population, most cervical lesions will subside naturally with the clearance of infection. The body's immunosuppression can increase the risk of HPV infection, such as immune system defect AIDS [5, 6]. There is a close relationship between HPV and cervical cancer. With the aggravation of pathological changes, the detection rate of HPV gradually increases. Therefore, some scholars put forward HPV testing as a screening method for cervical cancer.

RETRACTED

Early diagnosis is mainly through cytology, HPV detection, colposcopy, and biopsy. The diagnosis is mainly based on histological diagnosis. In addition, suspicious cases can also be found by ultrasound. Transvaginal ultrasound was used. During the examination, the probe slowly entered the vagina. The cervix was observed, including the size, echo, blood flow distribution, and its relationship with the surrounding, and then, the uterine body, intima, and accessories were examined [7, 8]. Ultrasonic elastography is a new type of ultrasonic diagnostic technology, which extracts the elastic characteristics of tissues and images them [9, 10]. In the ultrasonic diagnosis device, the starting receiving unit, A/D conversion module, and beam synthesis technology of the front-end system are accompanied by the image transmission module and operation. Therefore, the generated image also affects the doctor's diagnosis due to the influence of external noise [11–13]. van de Laar et al. [14] used linear region filtering to calculate the weighted average of the pixel points on the gray values or positional relationships of block pixels. Spatial filtering has a communication port. The size of the communication port determines the quality of related pictures nearby. The finer the pixels, the better the picture quality, which also determines the filtering effect. At present, the most commonly used bilateral filtering intelligent denoising algorithm can significantly improve the image quality when it is applied to ultrasonic elastography [15, 16].

RETRACTED

Therefore, in order to solve the problems of image noise, reduced resolution, and unclear image edge recognition in ultrasonic diagnosis, this study introduces the intelligent denoising algorithm of bilateral filter, which is applied to the elastic ultrasonic image of patients with CIN to denoise the image, so as to diagnose the disease. The purpose is to study the application value of ultrasonic elastography combined with HPV detection based on bilateral filtering intelligent denoising algorithm in the diagnosis of CIN.

## 2. Materials and Methods

### 2.1. Research Object and Grouping

This study selected 100 patients with cervical lesions treated in the hospital from September 2018 to September 2020 as the research object, including 50 patients with CIN and 50 patients with other lesions. There was no significant difference in clinical data between the two groups (*P* > 0.05), which was comparable. HPV detection was performed in 100 patients combined with ultrasonic elastography to diagnose cervical lesions. The experimental group used intelligent denoising algorithm to optimize the image map for diagnosis, while the control group did not use optimization. The differences between the two were analyzed and compared to analyze the application of ultrasonic elastography combined with HPV detection based on intelligent denoising algorithm in the diagnosis of CIN. This study was approved by ethics committee of hospital. The patients and their families understood the research contents and methods and agreed to sign the corresponding informed consent form.

Inclusion criteria are as follows: (1) aged between 18 and 65, (2) patients who can be diagnosed as cervical lesions after early clinical diagnosis, (3) patients did not receive other drug therapy recently during the study, (4) patients are willing to carry out this study, and (5) the study subjects had no other systemic diseases.

Exclusion criteria are as follows: (1) patients complicated with mental diseases or other systemic diseases, (2) persons suffering from reproductive system diseases, (3) incomplete clinical data, and (4) patients who did not fully cooperate with treatment due to personal factors.

### 2.2. Ultrasound Diagnosis

Patients were fasted and watered one night before ultrasound examination. Under fasting state, vaginal ultrasound examination was performed with vaginal color ultrasound examination instrument. The bladder lithotomy position was taken, and a certain amount of coupling agent was smeared on the top of the vaginal probe. The probe (ultrasonic probe frequency: 5-9 MHz, ultrasonic power: 3.5 W, scanning speed: 7 mm/s) was penetrated until the vaginal vault of the patient. Then, in order to obtain a clear image, the probe angle was adjusted accordingly, and the comprehensive scanning of the uterus, pelvis, and accessory structures was performed, including transverse, oblique, and longitudinal sections.

RETRACTED

The image of ultrasound examination in the experimental group was optimized by intelligent denoising algorithm, and the image noise and edge information were processed.

### 2.3. Intelligent Denoising Algorithm

Image noise will hinder people's understanding of the image. The purpose of denoising is to improve people's understanding of the image, and the purpose of denoising is to improve people's cognition of the image. Image denoising is conducive to further image processing, such as pixel enhancement and image edge detection. According to the influence on the signal, the noise model can be divided into additive noise and multiplicative noise. According to the principle of mean filter, a template is given; the mean value of all pixels in the template is used to replace the central pixel value of the original template [17, 18].

The main principle of bilateral filtering noise cancellation method is to use the weighted average of nearby pixels very similar to Gaussian convolution. The advantage of this algorithm is that it can smooth and maintain the flatness of the image edge considering the difference of gray value between the surrounding position points of the bilateral filter [19, 20]. To summarize the mechanism of bilateral filtering, the gray value of pixels depends on the gray value of surrounding pixels. It is necessary that two pixels are not only adjacent in spatial position but also have similar gray values. The bilateral filtering equation is as follows.

(1) $$\begin{array}{c} \text{BF}{\left[I\right]}_{P}=\frac{1}{w_{P}}\underset{q\in s}{\sum }G_{\sigma d}\left(\left\|p-\left.q\right\|\right.\right)G_{\sigma ,}\left(I_{p}-I_{q}\right)\cdot I_{q}. \end{array}$$

*W*_*P*_ is the normalization factor, and the equation is as follows.

(2) $$\begin{array}{c} w_{P}=\sum G_{\sigma d}\left(\left\|p-\left.q\right\|\right.\right)G_{\sigma r}\left(I_{p}-I_{q}\right). \end{array}$$

*σ*_*d*_ and *σ*_*r*_ are related to the image filtering value, and *G*_*σ*d_ further pixels can weaken the influence of noise, while the *G*_*σr*_ adjacent pixels can also weaken the influence of noise. Gaussian function is used to define *G*_*σd*_ and *G*_*σr*_; they are both spatial functions and functions to measure pixels. The equations are expressed as follows.

(3) $$\begin{array}{c} G_{\sigma d}=e^{-1/2{\left(d\left(p,q\right)/\sigma d\right)}^{2}},\\ G_{\sigma r}=e^{-1/2{\left(\sigma \left(I\left(P\right),I\left(q\right)\right)/\sigma \right)}^{2}}. \end{array}$$

*d*(*p*, *q*) is the linear distance between the two points on the image, *δ*(*I*(*p*), *I*(*q*)) is the pixel difference between the two points *p* and *q*, and this difference affects the denoising ability of bilateral filtering. The greater the *σ*_*d*_, the more blurred the image, and the same calculation method is used for *G*_*σr*_, so the more noise, the more blurred the image [21].

(4) $$\begin{array}{c} \text{SSIM}\left(x,y\right)=\frac{\left(2\alpha_{x}\alpha_{y}+c_{1}\right)\left(2\sigma_{xy}+c_{2}\right)}{\left(\alpha_{x}\alpha_{y}+c_{1}\right)\left({\sigma_{x}}^{2}+{\sigma_{y}}^{2}+c_{2}\right)},\\ \text{PSNR}=10\log_{10}\left(\frac{255^{2}\times M\times N}{\sum_{w=1}^{M}\sum_{e=1}^{N}\left|u\left(w,e\right)-f{\left(w,e\right)}^{2}\right.}\right). \end{array}$$

There are two ways for the noise reduction effect of images, namely, subjective evaluation and objective evaluation. The subjective evaluation is to observe the noise reduction effect with the human eyes, while the objective evaluation is shown by data. SSIM is the ratio of the same characteristics of the image structure, which can compare the quality and fineness of the image before and after compression [22, 23]. SSIM requires the simultaneous comparison of two graphs to calculate the identity and difference of the two graphs. The size of the image is set to *x* and *y*, and the equation is as follows.

(5) $$\begin{array}{c} \text{SSIM}\left(x,y\right)=\frac{\left(2\alpha_{x}\alpha_{y}+c_{1}\right)\left(2\sigma_{xy}+c_{2}\right)}{\left(\alpha_{x}\alpha_{y}+c_{1}\right)\left({\sigma_{x}}^{2}+{\sigma_{y}}^{2}+c_{2}\right)}. \end{array}$$

In the equation, the variance of pixels in the window is *σ*2, and C1 and C2 of Figure 1 represent the average gray value of pixels, namely, the dispersion of gray value of pixels in the image. The larger the SSIM value as the covariance of the image block *x* and *y*, the more similar the structural information between the noise removal image and the original image [24, 25]. Figure 1 shows the image denoising process.

RETRACTED

Peak signal to noise ratio (PSNR) is expressed as follows.

(6) $$\begin{array}{c} \text{PSNR}=10\log_{10}\left(\frac{255^{2}\times M\times N}{\sum_{w=1}^{M}\sum_{e=1}^{N}\left|u\left(w,e\right)-f{\left(w,e\right)}^{2}\right.}\right). \end{array}$$

*M* × *N* represents the size of the image. *u* and *f* are original and noise removal images. The higher the PSNR value, the better the image noise reduction effect [26].

### 2.4. Evaluation Indicators

The positive cases were patients with CIN, and the negative cases were patients with other lesions. True positive (TP) means that prediction is true. False positive (FP) means that the prediction is true and the actual is false. False negative (FN) indicates that prediction is false and actual is true. True negative (TN), prediction is false, actual is false. In this study, accuracy is used to represent the correct proportion of prediction, and the specific calculation method is expressed in Equation (7). Sensitivity (Se) represents the probability of positive cases being detected, which is expressed in Equation (8). Specificity (Sp) represents the probability of negative cases being detected, which is expressed in Equation (9).

(7) $$\begin{array}{c} \text{Accuracy}=\frac{\text{TN}+\text{TP}}{\text{TN}+\text{TP}+\text{FP}+\text{FN}}, \end{array}$$

(8) $$\begin{array}{c} \text{Se}=\frac{\text{TP}}{\text{TP}+\text{FN}}, \end{array}$$

(9) $$\begin{array}{c} \text{Sp}=\frac{\text{TN}}{\text{TN}+\text{FP}}. \end{array}$$

### 2.5. Statistical Methods

The data of this study was analyzed by the SPSS 19.0 statistical software, and the measured data was mean ± standard deviation (¯*x* ± *s*), and the count data was expressed in percentage (%). Analysis of variance was used for pairwise comparisons. The difference was statistically significant (*P* < 0.05).

## 3. Results

### 3.1. Image Processing Results

Figure 2 shows the image of cervical lesions of a random patient. The image shows that the cervix is significantly enlarged, the edge is not smooth, and the mucosal line is obviously bent or even interrupted. The echo of the whole uterine cavity is uneven, with multiple punctate and flake echo.

Figure 3 is the ultrasonic elastography of a random patient under the intelligent denoising algorithm. The cervix has increased irregularly, the edge contour is seriously deformed, and the cervical structure is also seriously deformed. The low echo area and uneven echo area account for the majority.

In Figure 4, Wiener filtering, mean filtering, and median filtering were compared with the intelligent denoising algorithm of bilateral filtering proposed in this research. It is found that the PSNR after Wiener filtering was the smallest, the PSNR after mean filtering and median filtering was slightly better, and the PSNR after intelligent denoising algorithm of bilateral filtering was the largest. Objectively, it was indicated that the algorithm proposed in this research was better than the traditional Wiener filter, mean filter, and median filter in filtering mixed noise.

### 3.2. Application of Ultrasonic Elastography Combined with HPV Detection Based on Intelligent Denoising Algorithm in the Diagnosis of CIN

Among cervical lesions, there were 50 cases of CIN and 50 cases of other lesions. HPV was detected in 100 patients combined with ultrasonic elastography. The experimental group used intelligent denoising algorithm to optimize the image map for diagnosis, while the control group did not use optimization. To evaluate three times, respectively, to improve the accuracy of the experimental results (Figure 5), in the experimental group, the average TP for three times is 94, the average FP for three times is 2, the average FN for three times is 6, and the average TN for three times is 98. In the control group, the average TP for three times is 96, the average FP for three times is 16, the average FN for three times is 14, and the average TN for three times is 84.

RETRACTED

Based on the above positive and negative cases, the indicators of the two groups were calculated (Figure 6). The three accuracy of the experimental group were 95%, 95%, and 98%, respectively; the three Se were 96%, 92%, and 94%, respectively; and the three Sp were 99%, 97%, and 98%, respectively.

The three accuracy of the control group were 84%, 86%, and 84%, respectively; the three Se were 88%, 84%, and 86%, respectively; and the three Sp were 81%, 83%, and 88%, respectively (Figure 7).

The average accuracy of the experimental group was 96%. The average accuracy of the control group was 85%. The accuracy of the experimental group and the control group was significantly different (*P* < 0.05) (Figure 8).

Figure 9 shows that the average Se of the experimental group was 94%. The average Se of the control group was 86%. There was significant difference in sensitivity between the experimental group and the control group (*P* < 0.05).

Figure 10 indicates that the average Sp of the experimental group was 98%. The average Sp of the control group was 84%. There was significant difference in specificity between the experimental group and the control group (*P* < 0.05).

## 4. Discussion

At present, relevant studies showed that the main ways of HPV infection and cervical lesions are sexual transmission and direct skin contact. The HPV infection rate of sexually active young women is the highest, and the infection rate decreases after the age of 30, but the risk of cervical lesions increases. In addition, the body's immunosuppression can increase the risk of HPV infection, such as immune system defects and AIDS. Different tissues in the human body have different elasticity due to different components. For example, in breast diseases, Smolarz et al. [27] found that there were significant statistical differences in hardness between normal and abnormal breast tissues, and the hardness of breast invasive ductal carcinoma was significantly higher than that of normal breast tissues. The traditional grayscale ultrasound image is based on the acoustic impedance difference of different tissues, while the elastic imaging image is based on the hardness difference of the object. The hardness difference between tissues is much greater than the acoustic impedance difference, and their difference is 104 times, which means that the imaging resolution of elastic imaging is much higher than that of traditional gray-scale ultrasound, which can diagnose diseases more sensitively.

RETRACTED

To analyze the application of ultrasonic elastography combined with HPV detection of intelligent denoising algorithm in the diagnosis of cervical intraepithelial neoplasia, 100 patients were tested for HPV by ultrasonic elastography. The experimental group used intelligent denoising algorithm to optimize the image for diagnosis, while the control group did not use optimization. The average values of TP, FP, FN, and TN in experimental group were 94, 2, 6, and 98, respectively. The average values of TP, FP, FN, and TN in the control group were 96, 16, 14, and 84, respectively. Based on the above positive and negative examples, the indexes of the two groups were calculated. The three-time accuracy rates of the experimental group were 95%, 95%, and 98%, respectively, while those of the control group were 84%, 86%, and 84%, respectively. The average accuracy rate of the experimental group (96%) was significantly higher than that of the control group (85%) (*P* < 0.05). The third sensitivity of the experimental group was 96%, 92%, and 94%, respectively, while that of the control group was 88%, 84%, and 86%, respectively. The average sensitivity of the experimental group (94%) was higher than that of the control group (86%), with significant difference (*P* < 0.05). The third specificity of the experimental group was 99%, 97%, and 98%, respectively, while that of the control group was 81%, 83%, and 88%, respectively. The average specificity of the experimental group (98%) was higher than that of the control group (84%), with significant difference (*P* < 0.05). The above data showed that the efficiency of ultrasonic elastography combined with HPV detection in the diagnosis of cervical intraepithelial neoplasia with intelligent denoising algorithm was higher than that without algorithm optimization, which was consistent with the research results of Wang et al. [28]. Then, the ultrasonic elastography of intelligent denoising algorithm was analyzed, and two experimental subjects were randomly selected. Patients in the control group underwent ultrasonic elastography without algorithm optimization, while patients in the experimental group underwent ultrasonic elastography optimized by intelligent denoising algorithm. By comparing the two images, it was found that the images optimized by intelligent algorithm were clearer and more distinguishable, which was helpful for doctors to diagnose and treat diseases.

RETRACTED

## 5. Conclusion

In this study, 100 patients with CIN were diagnosed by ultrasonic elastography combined with HPV detection. Aiming at the problems of noise, reduced resolution, and unclear image edge recognition of elastography, the intelligent denoising algorithm of bilateral filtering was proposed and applied to the image processing of elastography of CIN patients. The results show that the bilateral filtering intelligent denoising algorithm has a good denoising effect on elastic ultrasound images, and the ultrasound images processed by the algorithm combined with HPV detection have high accuracy in the diagnosis of CIN. However, there are few case samples selected in this study, which may have a certain impact on the experimental results, and the representativeness is low. Therefore, the sample size will be increased in the subsequent experiments to further study the diagnostic value of ultrasonic elastography combined with HPV detection for CIN. In conclusion, this study provides data support and theoretical basis for the diagnosis of CIN and other diseases.

## Figures and Tables

**Figure 1:** Ultrasonic image denoising process.

**Figure 2:** Ultrasound elastography without algorithm optimization in a random patient with uterine lesions.

**Figure 3:** Ultrasonic elastic image optimized by an intelligent denoising algorithm for a random patient with uterine disease.

**Figure 4:** Comparison of PSNR of four algorithms.

**Figure 5:** Data of positive and negative cases in the control group and the experimental group.

**Figure 6:** Data diagram of experimental group indicators.

**Figure 7:** Data graph of experimental group indicators.

**Figure 8:** Comparison of the average accuracy index between the experimental group and the control group. ^∗^ indicates that the accuracy of the experimental group was significantly different from that of the control group (*P* < 0.05).

**Figure 9:** Comparison of average sensitivity indexes between experimental group and control group. ^∗^ indicates that the accuracy of the experimental group was significantly different from that of the control group (*P* < 0.05).

**Figure 10:** Comparison of average specificity indexes between experimental group and control group. ^∗^ indicates that the accuracy of the experimental group was significantly different from that of the control group (*P* < 0.05).

## Data Availability

The data used to support the findings of this study are available from the corresponding author upon request.
